The article "Sylvian Fissure Lipoma: An Unusual Etiology of Seizures in Adults" was retracted in 2024. Reasons: false authorship; unreliable results or conclusions; no approval from an author; concerns about the authorship.

# Sylvian Fissure Lipoma: An Unusual Etiology of Seizures in Adults

**DOI:** 10.7759/cureus.21407

**Published:** 2022-01-19

**Authors:** Salihah M Ghazwani, Eman S Alzaki, Abdulaziz M Fadhel, Kholoud A Assiri, Lama W Alhabsi, Aishah M Babtain, Osama O Alkhudhair, Tharaa A Alanazi, Abdullah O Alsharif, Muhannad S Albadrani, Man K Alraddadi, Alaa A Alfayi, Meshal M Alsharari, Mohammed H Alruwaili, Faisal Al-Hawaj

**Affiliations:** 1 Medicine, King Khalid University, Abha, SAU; 2 Medicine, 6th of October University, 6th of October City, SAU; 3 Medicine, Umm Al-Qura University, Mecca, SAU; 4 Medicine, Jazan University, Jazan, SAU; 5 Medicine, Imam Mohammad Ibn Saud Islamic University, Riyadh, SAU; 6 Medicine, Tabuk University, Tabuk, SAU; 7 Medicine, Taif University, Taif, SAU; 8 Medicine, Taibah University, Medinah, SAU; 9 Medicine, Jordan University of Science and Technology, Irbid, JOR; 10 Medicine, Jouf University, Jouf, SAU; 11 Medicine, Imam Abdulrahman Bin Faisal University, Dammam, SAU

**Keywords:** case report, sylvian fissure, lipoma, magnetic resonance imaging, seizure

## Abstract

Seizure is a prevalent symptom and is an important neurological complaint in the emergency department. Patients with first-time seizures require a thorough evaluation to determine the possible etiologies and identify any causative pathology. Further, neuroimaging studies are vital to identifying the structural culprits. We report the case of a 35-year-old man who was brought to the emergency department with abnormal repetitive shaking movements that were witnessed by his spouse. Before the event, he became dizzy and fell to the ground. During the episode, he was not aware of his surrounding. He developed uprolling of his eyes and had frothy secretions from the mouth. On physical examination, the patient was drowsy but fully oriented. There were no signs of focal neurological deficit. Routine laboratory investigations, including hematological and biochemical profiles, yielded normal results. He was referred to undergo magnetic resonance imaging of the brain. The scan demonstrated the presence of a well-circumscribed lesion in the left Sylvian fissure with high signal intensity on T1- and T2-weighted image with suppression on the fat-suppressed sequence and no post-contrast enhancement. The radiological impression was of Sylvian fissure lipoma. The lesion was successfully resected surgically and the patient had an uneventful recovery with no complaints at the follow-up visits. Sylvian fissure lipoma is among the rarest locations of intracranial lipoma. Despite this, physicians should remember this lesion when they encounter a brain lesion with high signal intensity on T1- and T2-weighted images. While the majority of cases are incidental, an intracranial lipoma can be an etiology of first-time seizures in adults.

The article "Sylvian Fissure Lipoma: An Unusual Etiology of Seizures in Adults" was retracted in 2024. Reasons: false authorship; unreliable results or conclusions; no approval from an author; concerns about the authorship.

## Introduction

Seizure is a common neurological symptom with a reported lifetime prevalence of up to 10%. Further, seizures constitute 1% of the reasons to visit the emergency department [1]. Importantly, a significant proportion of these patients have a first seizure. Proper evaluation of patients with seizures is crucial. The first step is to recognize the seizure and differentiate it from other conditions that may mimic seizures, such as migraine and syncope. The etiology of seizures could be due to modifiable systemic derangements or an intrinsic brain pathology [2]. This will have a significant prognostic impact on the risk of having further seizures. Virtually, any cerebral insult could cause a seizure. The possible etiologies of seizures are broad and include a wide range of pathologies, such as ischemic or hemorrhagic stroke, traumatic brain insult, brain abscess, meningitis, and cerebral venous thrombosis [1]. Neuroimaging studies are vital to evaluate the culprit of structural cerebral lesions. Here, we present the case of a young man with a first-time seizure due to a Sylvian fissure lipoma.

## Case presentation

A 35-year-old man was brought to the emergency department by ambulance because he developed abnormal shaking movements. His spouse reported that they were having breakfast and suddenly he became dizzy and fell to the ground. Prior to that, he did not develop palpitation of chest pain. Further, he did not experience any abnormal sensations. During the episode, he was not aware of his surrounding. He developed uprolling of his eyes and had frothy secretions from the mouth. The abnormal repetitive movements involved his upper and lower extremities. Such movements were associated with urinary incontinence. After three minutes, the patient regained consciousness but appeared drowsy. This was the first episode of such movements. The patient had no significant past medical history. He was not on any medications. He did not have any history of smoking or alcohol drinking. The family history was non-contributory.

On physical examination, the patient was drowsy but fully oriented. There were no signs of focal neurological deficit. Both upper and lower limbs exhibited normal tone and power in the proximal and distal muscle groups. The coordination was intact. Further, examination of other systems showed normal results. Routine laboratory investigations, including hematological and biochemical profiles, yielded normal results (Table 1).

**Table 1:** Summary of the results of laboratory findings ESR: erythrocyte sedimentation rate; CRP: C-reactive protein

Laboratory Investigation	Result	Reference Range
Hemoglobin	14.5 g/dL	13.0–18.0
Leukocytes	6,800/mL	4.0–11.0
Platelet	440,000/mL	140–450
ESR	7 mm/hr	0–20
CRP	4.2 mg/dL	0.3–10.0
Total Bilirubin	0.7 mg/dL	0.2–1.2
Albumin	3.6 g/dL	3.4–5.0
Alkaline Phosphatase	49 U/L	46–116
Gamma-glutamyltransferase	22 U/L	15–85
Alanine Transferase	16 U/L	14–63
Aspartate Transferase	18 U/L	15–37
Blood Urea Nitrogen	11 mg/dL	7–18
Creatinine	0.8 mg/dL	0.7–1.3
Sodium	138 mEq/L	136–145
Potassium	3.6 mEq/L	3.5–5.1
Chloride	104 mEq/L	98–107

Since the patient did not have any previous history of seizures, he was referred to undergo magnetic resonance imaging of the brain. The scan demonstrated the presence of a well-circumscribed lesion in the left Sylvian fissure with high signal intensity on T1- and T2-weighted image with suppression on the fat-suppressed sequence and no post-contrast enhancement (Figures 1-3). The radiological impression was of Sylvian fissure lipoma.

The article "Sylvian Fissure Lipoma: An Unusual Etiology of Seizures in Adults" was retracted in 2024. Reasons: false authorship; unreliable results or conclusions; no approval from an author; concerns about the authorship.

**Figure 1:** Sagittal MR T1-weighted image showing a well-defined lesion (arrow) with high signal intensity seen in the left Sylvian fissure. MR: magnetic resonance

**Figure 2:** Axial MR T2-weighted image showing a well-defined lesion (arrow) with high signal intensity seen in the left Sylvian fissure. MR: magnetic resonance

**Figure 3:** Axial MR fat-suppressed image showing a well-defined lesion (arrow) with suppressed signal intensity in the left Sylvian fissure in keeping with lipoma. MR: magnetic resonance

Subsequently, the patient was referred to the neurosurgery team for further management. The patient underwent a left craniotomy. The mass lesion was removed from the Sylvian fissure. The patient had an uneventful recovery. Postoperatively, the patient was started on lornoxicam, levetiracetam, and dexamethasone. Histopathological examination confirmed the diagnosis of lipoma with the presence of mature adipose cells. The patient was discharged six days after the operation. At a two-year follow-up, the patient had no signs of recurrence or new symptoms.

## Discussion

We reported the case of an intracranial Sylvian fissure lipoma presenting with a seizure in a young adult. Intracranial lipoma is a rare benign tumor of adipose cells having an incidence of 0.08% in the postmortem examination studies [3]. Further, a retrospective study involving 3,000 patients with head computed tomography scans performed for patients with trauma yielded only three cases of lipoma [4]. Such tumors are typically found incidentally and receive conservative management. However, Sylvian fissure lipoma is among the rarest sites of intracranial lipoma [5].

Regarding the pathogenesis of intracranial lipoma, it is thought that the lipoma develops because of abnormal differentiation of the mesenchymal covering of the brain, which is termed the meninx primitiva. Considering this hypothesis, it is not unexpected to see associated congenital brain malformations in patients with intracranial lipoma. Indeed, it is reported that over 50% of patients with intracranial lipoma have associated a wide range of anomalies, including corpus callosum agenesis, cortical dysplasia, neural tube defect, encephalocele, and hypoplastic vermis [6]. In the present case, however, the finding of Sylvian fissure lipoma was isolated with no associated anomalies.

The article "Sylvian Fissure Lipoma: An Unusual Etiology of Seizures in Adults" was retracted in 2024. Reasons: false authorship; unreliable results or conclusions; no approval from an author; concerns about the authorship.

Intracranial lipoma can be diagnosed with high accuracy using neuroimaging studies with computed tomography or magnetic resonance imaging. The computed tomography scan demonstrates a well-circumscribed lesion with homogeneous fat-attenuation that can show calcification but has no post-contrast enhancement. In magnetic resonance imaging, the lesion demonstrates high signal intensity on the T1- and T2-weighted images that are suppressed on fat-saturated sequences [6]. The most important differential diagnosis of intracranial lipoma is a dermoid cyst. However, the latter exhibits a heterogeneous appearance due to its various components. Additionally, the dermoid cyst tends to displace rather than encase the surrounding structures [7].

## Conclusions

Sylvian fissure lipoma is among the rarest locations of intracranial lipoma. Despite this, physicians should remember this lesion when they encounter a brain lesion with high signal intensity on T1- and T2-weighted images. While the majority of cases are incidental, an intracranial lipoma can be an etiology of first-time seizures in adults. Careful radiological evaluation of patients with Sylvian fissure lipoma is needed because of the associated congenital malformation.
